The article "The Effect of Qingre Huayu Recipe on Wound Healing after Anal Fistulotomy in Sprague-Dawley Rats" was retracted in 2023. Reasons: unreliable results or conclusions; concerns about the data; concerns about the peer review; concerns about the citations.

# The Effect of Qingre Huayu Recipe on Wound Healing after Anal Fistulotomy in Sprague-Dawley Rats

**DOI:** 10.1155/2022/9397478

**Published:** 2022-04-19

**Authors:** Jiazhi Gao, Jiandong Wang, Ping Chen, Peilin Ding, Liang Tian, Biao Liang, Zhan Shi

**Affiliations:** Department of Proctology, Putuo Hospital, Shanghai University of Traditional Chinese Medicine, No. 164 Lanxi Road, Shanghai 200333, China

## Abstract

Anal fistula is a common anorectal disease. At present, most scholars believe that its pathogenesis is related to anal gland infection. Anal fistula cannot heal on its own after the onset and must be treated surgically. The wound of anal fistula surgery is open and polluted, and it belongs to three types of three-stage healing; it is the most difficult to heal among all surgical incisions, with a long course of disease, a lot of exudation, and pain for the patient; traditional Chinese medicine has rich experience in the treatment of postoperative wound healing of anal fistula. The study aimed to evaluate the mechanism of Qingre Huayu (QRHY) Recipe on wound healing after fistulotomy on SD rats. SD rats (*n* = 72) were randomized into three groups post-anorectal surgery. The rats in the positive control group were given potassium permanganate (PP), treatment group were given QRHY, and trauma model group were given 0.9% normal salinity. The changes in wound secretion, granulated tissue, and epithelium tissue were observed, and wound healing rates were evaluated by the discrepancies in wound area. HE and Masson's staining as well as transmission electron microscopy were also performed. The localization as well as the measurement of Ang1, Src, and VE cadherin expression in each group adopted real-time PCR, western blot, and immunohistochemistry (IHC) assays. Statistically higher wound healing rates were observed in QRHY group on days 3, 7, and 14 compared with other groups. Histological analyses showed highly significant increase in collagen and fibroblasts, less inflammatory cells, and vascular endothelial permeability in QRHY rats. The transmission electron microscopy revealed that the intact structure of tight junctions in endothelial cells and well-organized collagen and VE-cadherin, Ang1, and Tie-2 were upregulated by QRHY, while Src was inhibited. This study showed that QRHY can promote wound healing after anal fistulas.

## 1. Introduction

Anal fistula, an abnormal passage connecting the anorectal mucosa to the external skin and occur de novo or after acute anorectal abscess, is a common surgical approach with high incidence and causes pain to patients [1]. In surgery, the current mainstay of treatment for anal fistula is difficult to eliminate potential postoperative risk factors like long wound healing time and susceptibility to infection [2]. Hence, the shortening postoperative wound healing is an urgent issue to be solved clinically.

Local inflammation response, granulation tissue (GT) formation, and tissue reconstruction, the three main processes of wound healing, determine the duration and quality of healing [3]. As the main cellular constituents, GTs and fibroblasts (FBs) are essential in wound healing [4]. Reportedly, treating wounds with traditional medicinal remedies is a vital means to accelerate wound healing. Experimentally, some plants and herbs have been used as traditional medicine to treat wounds and achieved encouraging outcomes [5, 6].

After long-term clinical observation and literature review, from the perspective of the entire course of anal fistula surgery, traditional Chinese medicine believes that the wound healing process after anal fistula surgery is not only manifested in “hot” symptoms such as “redness, swelling, heat, and pain”, but also “heat” symptoms. The skin around the wound is moist, the wound exudates, the pus is thick, and the granulation tissue is reddish. The pathogenesis of postoperative wound symptoms is mainly caused by “damp heat”. The Qingre Huayu (QRHY) Recipe for clearing heat and removing blood stasis is composed of *Sophora flavescens*, treats, frankincense, and myrrh and has the functions of clearing away heat and removing dampness, promoting blood circulation and relieving pain, reducing swelling, and promoting muscle growth. The antiinflammatory, antiallergic, liver protection, and diuretic effects of *Sophora flavescens* in the prescription are the performance of *Sophora flavescens* for clearing away heat and dampness [7]. *Phellodendron* has the functions of clearing heat, drying dampness, purging fire, and detoxification. Pharmacological studies have also proved that *Phellodendron* has a certain relaxation effect on some striated muscles, which can reduce the pressure of the anal canal, improve the local circulation of the anal canal, and promote wound healing [8–10]. Frankincense has the effects of regulating qi and promoting blood circulation, calming pain, and chasing poison. Modern pharmacological research shows that frankincense has antiinflammatory and antitumor effects [11]. It has anti-inflammatory and analgesic effects in pharmacological [12]. The compatibility of the above medicines can be said to complement each other and bring out the best in each other.

The wound of anal fistula surgery is open and polluted, and it belongs to three types of three-stage healing; it is the most difficult to heal among all surgical incisions, with a long course of disease, a lot of exudation, and pain for the patient; traditional Chinese medicine has rich experience in the treatment of postoperative wound healing of anal fistula. The patients with anal fistula have obvious advantages in terms of clinical symptoms and promoting wound healing. In the process of wound healing, inflammation always accompanies. Moderate inflammation promotes healing, while excessive inflammation delays healing. In the past, most studies have been conducted from the aspect of growth factors, mainly focusing on the later stage of wound healing. The Qingre Huayu Recipe starts from the relationship between vascular permeability and inflammation and explores its mechanism of promoting wound healing.

However, there is a paucity of studies on the effects of traditional Chinese medicines, including *Sophora flavescentis radix*, *Phellodendron amurense Rupr*, *Boswellia*, and *Commiphora myrrha*, on wound healing, which needs an in-depth study.

## 2. Materials and Methods

### 2.1. Postanal Fistula Wound Healing Model

Totally 72 male SD rats weighing 250 ± 20 g from Shanghai Laboratory Animal Center CAS (Shanghai SLAC Laboratory Animal Co., Ltd, Shanghai, China) had access to tap water and standard rat chow. After two weeks, all animals were randomized into the QRHY treatment group (*n* = 24), PP control group (*n* = 24), and 0.9% normal salinity group (*n* = 24). The method of Recknagel et al. [7] was used with slight modification. After hair removal with 8% Na2S for 3 days, the rats were anesthetized with 2.5% sodium pentobarbital (30 mg/kg) (sigma, USA) [13], and their preparation area was sterilized by 0.1% tincture of bromogeramine, and then a circular incision with 2 cm diameter was made on the buttocks of the rats from the skin, and fascia to the surface of the muscle was excised entirely. After hemostasis, the rats were fed without bandaging to cause infection similar to postclinical anal fistula surgery. The ethics committee at the Putuo Hospital, Shanghai University of Traditional Chinese Medicine approved this study without reserves. All the protocols were in conformity with declaration of Helsinki. The modeling method of this experiment was improved by referring to the modeling methods of Fu Xiaobing [14], Dong Qingjun [15], and Zheng Xueping [16].

#### 2.1.1. Growth of Granulation Tissue

In the morning on the 3rd, 7th, and 14th postoperative days of the growth of granulation tissue was recorded when dressinsg was changeds in the morning condition. The specific scoring standard is as follows: 0 point, where the wound surface is smooth, the granulation is vigorous and long, and the color is red; 1 point, where the wound surface is flat and uniform, the granulation is more vigorous, and the color is pale red; 2 points, where the wound surface is not flat, the granulation grows slowly, and it has a pale color; and 3 points, where the the wound surface is sunken, the granulation growth is not obvious, and the color is dull.

#### 2.1.2. Exudation of Wound Secretions

The exudation of wound secretions was recorded in the morning on the 3rd, 7th, and 14th postoperative days when dressing was changed. The specific scoring criteria is as follows: 0 point, where the wound is bright red with no obvious secretions; 1 point, where the amount of secretions is small and one piece of gauze is not penetrated gauze; and 3 points, where there is a large amount of secretions that penetrate 2 or more pieces of gauze.

### 2.2. Drugs and Instruments

The QRHY was composed of *Sophora flavescentis radix* (30 g), *Phellodendron amurense Rupr* (20 g), *Boswellia* (20 g), and *Commiphora myrrha* (20 g), and the fumigation solution was provided by Shanghai Putuo District Central Hospital Pharmacy, and the decoction : water ratio was 1 : 9. Potassium permanganate (PP) and saline were provided by the Jinan Kangfusheng Manufacturing Co., Ltd. (JiNan, China). An electric constant temperature water tank was provided by the Shanghai Shengke Instrument Equipment Co., Ltd. (Shanghai, China). The traditional Chinese medicine prescriptions (30 g of *Sophora flavescens*, 20 g of treats, 20 g of frankincense, and 20 g of myrrh) were added to 1000 ml of cold water and soaked for 45 minutes. Decoct at low heat for about 30 minutes, decoct 250 ml of medicinal liquid, add about 750 ml of water to the medicinal residue, decoct 250 ml as above, mix the medicinal liquid twice, pour the medicinal liquid into the fumigation and washing machine during fumigation and wash, and keep the medicinal liquid at a constant temperature of 40 °C Fumigate for 20 minutes.

### 2.3. Treatment with QRHY after Anal Fistulotomy

24 h after anal fistulas, the experimental rats were treated with QRHY, while the control rats were treated with the same quantity of PP or saline baths twice a day for 20 min. The solution was applied 3 cm from the wound, and the wire cage was placed in a 40 °C electric water bath and 40 °C constant temperature liquid fumigation for 20 minutes.

### 2.4. Wound Healing Rates

The area of wound was determined by Image J in each group on the 0, 3^rd^, 7^th^, and 14^th^ postoperative days, respectively. Wound healing rate = (the area on the first day after the operation - the area on the day of the photo) / the area on the first day after the operation × 100% (Senthil Kumar et al., 2006).

### 2.5. Histological Analysis

Granulated tissues were collected on the 3^rd^, 7^th^, and 14^th^ days after anal fistulotomy after anesthesia by ketamine (15 mg/100 g) (sigma, USA) and then fixed in 10% neutral buffered formalin (NBF). The tissues fixed in formalin were subjected to dehydration through grades of alcohol, xylene clearing, and subsequent paraffin-embedding (58–60°mp). Thereafter, the samples were stained with hematoxylin and eosin (H&E) before the wound tissue edemas, GT hyperplasia, inflammatory cell infiltration, and wound healing were observed in each group, respectively. Meanwhile, the synthesis and distribution of collagen were observed with Masson's trichrome staining [8].

### 2.6. Transmission Electron Microscopy (TEM)

The wounded tissues were divided into smaller pieces and collected on the 0, 3^rd^, 7^th^, and 14^th^ postoperatively for fixation in 5% glutaraldehyde. Then, the fixed tissues were processed for postfixation (2 h) (Sinopharm Group, china) in 1% osmium tetroxide (OsO4), dehydration through graded acetic acid and propanol, and resin-embedding to obtain ultrathin section in copper grid. Then, the staining with uranium acetate and lead citrate was done. The synthesis and distribution of the tightly connected vascular endothelial cells and collagen fiber were made with the use of a transmission electron microscope (Tecnai G2 Spirit Bio TWIN).

### 2.7. Vascular Permeability

Granulated tissues, collected on the 0, 3rd, 7th, and 14 th postoperative days, were stained by Evans Blue and then dissolved in formamide (2 mL) for 48 h at room temperature. The permeability of newly formed capillaries was investigated by enzyme-labeled instrument under 420 nm [9].

### 2.8. Real-Time PCR

The tissues, stored at –80°C immediately after collection on the 3^rd^, 7^th^, and 14^th^ postoperative days, were disrupted by manual pestle grinding to prepare tissue homogenate. Trizol-isolated total RNA from tissue homogenate was detected by detected by agarose electrophoresis and NanoDrop 2000 (Thermo Scientific, USA) and then reverse-transcribed to cDNA (Takara Biomedical Technology, China). Next, the qPCR reactions were performed based on the following conditions: predenaturation cycle for 20 s at 95 °C, annealing cycle for 30 s at 58 °C, and 40 extension cycles for 30 s at 72 °C. The internal control was *β*-actin and the 2−*ΔΔ*Ct method for computing the relative mRNA expression. The primer sequences were listed as follows: Src F: (5′-to-3′;): TGGCGAGAACCTGGTGTGCAA, R (5′-to-3′): TTGGCACCTTGCCGAGCTGTT; VE-cadherin F (5′;-to-3′): ACCTCATCACCTTGGGTAGC, R (5′-to-3′): CCAGACAGAACACCATCCTG; Ang1 F (5′-to-3′): CACCAACAACAGTGTCCT, R (5′-to-3′): CTTCCTCTCTTTTTCCTCC; and Tie2 F (5′-to-3′): CCTTCACCAGG CTGATTGTT, R (5′-to-3′): AATGCATTCCCCGGTATCTT.

### 2.9. Western Blotting

After excessive anesthesia in rats leading to death, the tissue of wound was collected. Total protein was extracted, and after the determination of its concentration by bicinchoninic acid (BCA) assay (Pierce, Rockford, IL, USA), the protein was treated with 10% sodium dodecyl sulfate-polyacrylamide gel electrophoresis (SDS-PAGE) separation as well as transferred onto a nitrocellulose membrane. Src (ab133283, ABCAM, USA,1 : 2000), VE-cadherin (ab231227, ABCAM, USA,1 : 5000), Ang1 (ab133425, ABCAM, USA,1 : 5000), Tie-2 (19157-1-AP, Proteintech, USA,1 : 5000), and *β*-actin (ab8226, ABCAM, USA,1 : 5000) antibodies were added for incubation overnight at 4 °C. Then came the indoor cultivation (1 h) with the corresponding II antibodies. Enhanced chemiluminescence (Thermo Fisher Scientific, Waltham, MA, USA) was carried out, and Fluor Chem 2.0 image analyzer was applied to analyze.

### 2.10. Immunohistochemistry

The expression of Src, VE-cadherin, and Ang1 was analyzed using immunohistochemistry. Paraffin specimens were made into 3-*μ*m-thick slices, dewaxed in xylene and subjected to hydration in ethanol gradient. After blocking endogenous activity with 0.3% H_2_O_2_, the slices were cultivated with serum for 1 h at ambient temperature to block nonspecific staining. With the use of a Histomouse Max broad spectrum 3,3-diaminobenzidine (DAB) kit (Invitrogen), the slices were then immunostained with Src, VE-cadherin, Ang1, and Tie-2. Slide scanning was performed using a Leica SCN400 slide scanner with the aid of image viewer software.

### 2.11. Statistical Processing

The results are presented as the mean ± SD. One-way or two-way ANOVA with subsequent Dunnett's multiple comparisons posttest were performed for comparisons between 3 or more groups. Student's *t*-test was carried out for comparisons among two groups. GraphPad Prism Software (version 8.0; GraphPad Software, La Jolla, California) and SPSS 21 (IBM, USA) were used for the analysis. *P* < 0.05 was considered to indicate statistical significance.

## 3. Results

### 3.1. Assessment of In Vivo Wound Healing Activity

*In vivo* experiments were conducted to reveal the wound healing effect of QRHY. The number of rats with wound secretion, tissue edema, and inflammation is shown in Tables 1–3 after 3, 7, and 14 days. The salinity and PP group showed wound secretion, tissue edema, and inflammation on the wound after the 3-day treatments. The changes observed in salinity group and PP group were inhibited by QRHY treatment (Table 1). After the 7- and 14-day treatments (Tables 2 and 3), the wounds of rats in all groups were repaired to a large extent including epithelium tissue repair and GT formation. Wound healing was noted in QRHY group without wound secretion, tissue edema, or inflammation compared to salinity and PP groups with lesser wound secretion and inflammation. Furthermore, the photographs of wound treated with QRHY, PP, or 0.9% normal salinity for 3, 7, and 14 days are shown in Figure 1 and indicated that QRHY group exhibited an excellent healing effect after 3 and 7 days, compared to the PP and salinity group. Two weeks later, the wound healing in QRHY and PP groups reached nearly 95%, versus the salinity-treated group (Figure 1, Table 4).

### 3.2. Histological Analysis

Wound healing including the phasesis of hemostasis, inflammation, migration, proliferation, and maturation [10] is a complex biological process associated with tissue regeneration. In this study, the progress of wound healing was evaluated by H&E staining. As shown in Figure 2, inflammatory cells emerged after treatment with the salinity and PP group for 3 days, while some FBs and immature glandular cavity was observed in QRHYs group. QRHY group had less residual inflammatory cells on the wound than salinity and PP groups 7 days posttreatment. Besides, the PP and salinity group produced microvessels and some FBs, while mature glands were observed in QRHYs group under the same conditions. After 14 days of treatment, less inflammatory cells were found on the wound after PP treatment compared to salinity treatment. Meanwhile, the wound epidermis in the PP group was incomplete, thinner, and intact, while the thickening of the epidermis was observed in QRHY rats. The extent of collagen deposition was detected by histomorphometry on sections stained with Masson (Figure 3). By 14 days of healing, collagen deposition was enhanced on wound healing by treatment with QRHY, compared to the saline and PP-treated group which showed the lack of collagen. There was complete re-epithelialization in QRHY group after 14-days. It showed that QRHY can accelerate epithelial crawling and GT proliferation to promote wound healing. Therefore, we concluded that QRHY exhibited the best wound healing effect.

### 3.3. TEM

TEM confirmed the presence of microvascular endothelial cells and the distribution of collagen fibers (Figure 4). Collagen fibers filled the lacunae 14 days posttreatment. The collagen fibers showed disorganization in salinity group, while they showed a clear orientation and miniature gaps between fibers after PP treatment for 14 days. At the end of QRHY treatment for 14 days, there was no lacuna and collagen fibers were almost normally organized. Meanwhile, the ultrastructure of microvascular endothelial cells was observed under TEM, and it was found that QRHY could change the open state of tight junctions between endothelial cells and restore the intact structure of tight junctions after 14d, prompting that QRHY may influence tight junctions between endothelial cells and lower vasopermeability.

### 3.4. The Influences of QRHY on Vascular Permeability in Wound Healing after Anal Fistulas

3, 7, and 14 days after QRHYs treatment on wound healing, the vascular permeability was assessed by Evans blue staining (Table 5). The permeability of blood vessels in 0.9% salinity group was significantly higher than QRHY group and PP at 3, 7, and 14 days (P < 0.05). There was no statistical difference between the QRHY and PP groups (P > 0.05). The permeability of blood vessels in the QRHY group was significantly decreased (to 28.43 ± 5.30) when compared with the PP group (P < 0.05) at 14 days. These findings indicated that QRHY can significantly decrease vascular permeability in wound healing after anal fistulas.

### 3.5. Effect of QRHY Treatment on Src, VE-Cadherin, Ang1, and Tie-2 mRNA Expression in Wound Healing after Anal Fistulas in Rats

RT-qPCR was used to detect the effect QRHY on the expression levels of tight junction-associated proteins Src, VE-cadherin, Ang1, and Tie-2 mRNA at 3 d, 7 d, and 14 d after anal fistulas (Figure 5(a)). The expression levels of VE-cadherin, Ang1, and Tie-2 mRNA levels were significantly increased in PP and QRHY groups compared to saline group (Figure 5(a)). However, Src mRNA was inhibited by the treatment with either PP or QRHY (Figure 5(a)). The alterations of Src, VE-cadherin, Ang1, and Tie-2 protein levels on the 3^rd^, 7^th^, and 14^th^ days of wound healing after anal fistula were measured by western blotting (Figure 5(b)). The expression level of the Src protein in rats in PP and QRHYs groups was significantly decreased compared to the saline group, while the expressions of VE-cadherin, Ang1, and Tie-2 protein in rats in QRHY group were significantly increased compared to other groups on the 3^rd^, 7^th^, and 14^th^ days (Figure 5(b)). The visualization of subcellular localization of Ang1, Src, and VE-cadherin in GTs adopted IHC (Figure 6). In rats, Ang1, Src, and VE-cadherin protein were present in cytoplasmic, and no difference was observed between the three groups after anal fistulas for 3d. QRHYs treated rats showed strong, positive cytoplasmic Ang1 and VE-cadherin staining, whereas less cytoplasmic expression of localized Src was observed compared to PP rats after 14 days.

## 4. Discussion

Anal fistula is a common anorectal disease with high incidence and causes suffering to patients; the most frequently used therapy for this condition is surgery [17, 18]. Most of the wounds left after the operation are open wounds. On the one hand, the surgical incision is open and polluted, and it belongs to the three types of three-stage healing, which is the most difficult to heal among all surgical incisions. Furthermore, the healing of wounds is slow because of infections, pain, and lack of blood. Therefore, strategies for improved wound healing after anal fistula are urgently needed. The traditional Chinese medicine (TCM) plays an important role in maintaining people's health with its reliable therapeutic efficacy and fewer side effects [19]. In recent years, fumigation-washing therapy of surgical wounds by herbal fumigant has been widely used for postoperative treatment with satisfactory results [20]. In this study, the effect of QRHY on wound healing after anal fistula was explored. We found that QRHYs significantly reduced inflammatory cells and restored the well-organized structure of collagen and fibroblasts in rats. Furthermore, we observed the intact structure of tight junctions in endothelial cells and significant decrease of vascular endothelial permeability upon QRHY treatment. Meanwhile, the increased expression levels of VE-cadherin, Ang1, and Tie-2 and decrease level of Src were also found in QRHY-treated rats. These results suggested that QRHY might have therapeutic effects in wound healing after anal fistulas.

Wound healing involves multiple cooperative molecular processes including inflammation, angiogenesis, wound contraction, granulation tissue formation, and re-epithelialization [21]. Therefore, it is possible to judge the effect of QRHY fumigation therapies on wound healing by observing wound healing at different time points in rats. In this study, significant wound healing was observed in QRHYs treated rats. *In vivo* epithelialization of rats supports the effect of QRHY in wound healing. Significant reduction of infiltrating inflammatory cells and increase of early dermal and epidermal regeneration by histological examinations was observed, which further confirmed the therapeutic effect of QRHY.

Previous studies showed that wound contraction, an essential phenomenon in the process of healing, is mediated by the differentiation of fibroblasts into myofibroblasts within granular tissue. Thus, the presence of myofibroblasts during wound healing is considered an important feature of tissues to undergo contraction [22–24]. The researchers previously reported that the hesperidin treatment can enhance wound healing in nondiabetic rats by increased fibroblasts proliferation [25]. In this study, the quick rate of wound healing in QRHY rats may be attributable to the presence of enhanced proliferation of fibroblasts, which promoted wound contraction. Furthermore, TEM images showed that QRHYs could change the open state of tight junctions between endothelial cells and restore the intact structure of tight junctions and collagen fibers in wound healing after anal fistulas. The highly significant increase of collagen revealed the enhanced migration of fibroblasts, epithelial cells, and synthesis of extracellular matrix including collagen during the healing process in QRHYs rats [8]. Here, we speculated that the increased collagen in QRHYs rats may be a result of enhanced proliferation of fibroblast leading to wound healing.

Vascular permeability plays a key role in wounds healing of skin [26]. The phosphorylation of VE-cadherin mediated by Src in permeability has been studied extensively. The role of SRC activity in the regulation of endothelial permeability was reported previously. Transient activation of SRC reduced the endothelial permeability due to VE-cadherin phosphorylation on Y731 [27]. Therefore, the role of Src/VE-cadherin signaling pathways in vascular permeability has received much attention. In this study, the reduction in the permeability was accompanied with decreased Src and increased of VE-cadherin expression levels in QRHYs rats. Our study suggested that SRC-mediated phosphorylation of VE cadherin contributes to reducing endothelial permeability to promote wound healing.

The Src/VE-cadherin signaling pathway is a biologically efficient cellular signal transduction pathway that is regulated by multiple cytokines, including vascular endothelial growth factor (VEGF) and angiopoietin I (Ang I) [28]. Ang-1, acting as a ligand of the Tie receptor tyrosine kinase, is a type of 70 kDa glycoprotein from angiopoietin family [2519]. Tie-2, as a regulator of integrins, is essential for the maintenance of the integrity and function of tissues in adults [29]. Previous studies showed the acceleration of wound healing through angiogenesis after application of recombinant adenovirus encoding angiopoietin-1 (Ad-Ang-1). Thus, a substrate with the ability to activate Ang-1-Tie signaling may serve as an effective therapeutic candidate for angiogenesis and vascular protection [30]. In this study, the upregulation of Ang-1-Tie can result in an increased angiogenesis, hence accelerating wound healing via stabilized blood vessel integrity and vascular remodeling after treatment with QRHYs rats.

Recently, QRLSs have been reported effective in dealing with wound healing [31]. In addition, herbal formulae showed its wound healing potential against chronic diabetic ulcers [32]. These results provided evidence for using natural medicines such as QRHYs in wound healing.

In conclusion, the results of the present study showed that QRHY can increase Ang-1 and Tie2 levels resulting in increased angiogenesis and VE cadherin via SRC activation, which contributes to decreased vascular endothelial permeability and promoted wound healing.

## Figures and Tables

**Figure 1:** Photographs of wound healing *in vivo*.

**Figure 2:** Photomicrographs of hematoxylin and eosin (H&E) stained tissues. The progress of wound healing was evaluated by H&E staining (×40 magnification, scale bar = 50 *μ*m).

**Figure 3:** Photomicrographs of Masson-stained tissues. The extent of collagen deposition was detected with Masson stained (×40 magnification, scale bar = 50 *μ*m).

**Figure 4:** Ultrastructure analysis by transmission electron microscopy. Tight junctions of vascular endothelial cells and collagen were observed under TEM in wound healing. The microvascular endothelial cells and the distribution of collagen fibers were observed after treatment for 14 days (×5000 magnification and ×10000 magnification).

**Figure 5:** mRNA and protein expression analysis. (a) Quantitative representation of expression of Src, VE-cadherin, Ang1, and Tie-2 mRNA were evaluated. (b) Western blotting showing the expressions of Src, VE-cadherin, Ang1, and Tie-2 protein and corresponding semiquantitative analysis of protein level of Src, VE-cadherin, Ang1, and Tie-2. Data are expressed as mean ± SEM (n = 3) and analyzed by one-way ANOVA, P < 0.05. Data are expressed as mean ± SEM (n = 3) and analyzed by one-way ANOVA.

**Figure 6:** Immunohistochemical analysis (IHC) on granulation tissue of rats showing the changes of Ang1, Src, and VE-cadherin expression. IHC (×40 magnification, scale bar = 50 *μ*m) was performed on rats showing Ang1, Src, and VE-cadherin expression with treatment after anal fistulas for 3, 7, and 14 days.

**Table 1:** Visual observation of wound healing after 3 days.

	*n*	Granulation tissue		Epithelium tissue		Wound secretion			
		Yes	No	Yes	No	-	+	++	+++
QRHYs	24	14	10	10	14	3	8	7	6
PP	24	9	15	3	21	2	5	8	9
0.9% salinity	24	4	20	1	23	0	5	9	10

- means 0 points, + means 1 point, ++ means 2 points, +++ means 3 points.

**Table 2:** Visual observation of wound healing after 7 days.

	n	Granulation tissue		Epithelium tissue		Wound secretion			
		Yes	No	Yes	No	-	+	++	+++
QRHYs	24	16	8	15	9	13	7	4	0
PP	24	9	15	8	16	6	9	4	5
0.9% salinity	24	7	17	7	17	5	8	6	5

- means 0 points, + means 1 point, ++ means 2 points, +++ means 3 points.

**Table 3:** Visual observation of wound healing after 14 days.

	n	Granulation tissue		Epithelium tissue		Wound secretion			
		Yes	No	Yes	No	-	+	++	+++
QRHYs	24	23	1	23	1	22	2	0	0
PP	24	22	2	21	3	19	4	1	0
0.9% salinity	24	21	3	21	3	17	5	1	1

- means 0 points, + means 1 point, ++ means 2 points, +++ means 3 points.

**Table 4:** Wound healing rate after anal fistulas (%) (X ± SD).

	*n*	3 days	7 days	14 days
QRHYs	24	22.49 ± 4.31^∗∗^	55.05 ± 5.21^∗∗^	96.42 ± 0.64
PP	24	18.72 ± 6.08^∗^	50.87 ± 5.78^∗∗^	90.08 ± 0.55
0.9% salinity	24	11.54 ± 6.38	38.48 ± 7.59	85.62 ± 1.24

∗*P* < 0.05 VS 0.9% salinity; ∗∗*P* < 0.01 VS 0.9% salinity.

**Table 5:** Neovascular permeability detected by Evans blue dye (EBD) injection.

	*n*	3 days	7 days	14 days
QRHYs	24	41.35 ± 5.17^∗^	33.73 ± 7.82^∗∗^	28.43 ± 5.30^∗∗^
PP	24	40.15 ± 8.33^∗^	29.60 ± 5.25^∗∗^	223.84 ± 4.14^∗∗##^
0.9% salinity	24	55.85 ± 8.70	65.75 ± 7.69	66.49 ± 7.12

∗*P* < 0.05 VS 0.9% salinity; ∗∗*P* < 0.01 VS 0.9% salinity. ^##^*P* < 0.01 VS QRHYs.

## Data Availability

The simulation experiment data used to support the findings of this study are available from the corresponding author upon request.
